RETRACTED

# MicroRNA-506 inhibits tumor growth and metastasis in nasopharyngeal carcinoma through the inactivation of the Wnt/β-catenin signaling pathway by down-regulating LHX2

**DOI:** 10.1186/s13046-019-1023-4

**Published:** 2019-02-21

**Authors:** Tian-Song Liang, Ying-Juan Zheng, Juan Wang, Jing-Yi Zhao, Dao-Ke Yang, Zhang-Suo Liu

**Affiliations:** Department of Radiotherapy, the First Affiliated Hospital of Zhengzhou University, Zhengdong Branch, Zhengzhou, 475000 Henan Province People’s Republic of China

**Keywords:** MicroRNA-506, LIM Homeobox 2, Wnt/β-catenin signaling pathway, Epithelial-mesenchymal transition, Lymph node metastasis, Nasopharyngeal carcinoma

## Abstract

**Background:**

Epithelial-mesenchymal transition (EMT)-associated proteins play key roles in cancer progression and metastasis with the involvement of microRNAs (miRNAs). This study aims to assess the role of miR-506 working in tandem with LIM Homeobox 2 (LHX2) in EMT and metastasis through the Wnt/β-catenin signaling pathway in nasopharyngeal carcinoma (NPC).

**Methods:**

Differentially expressed genes associated with NPC were screened using microarray analyses, from which LHX2 was identified. Next, the potential relationship between miR-506 and LHX2 was analyzed. In order to explore the effect of miR-506 or LHX2 on NPC cell proliferation, migration, invasion and apoptosis, serials of mimics, inhibitors or siRNA against LHX2 were transfected into NPC cells. Then, the expression patterns of LHX2, Wnt1, β-catenin, E-cadherin, Vimentin, TCF4 and Twist were determined to assess the influence of miR-506 or LHX2 on EMT as well as the relationship between the Wnt/β-catenin signaling pathway and TCF4. The tumorigenicity and lymph node metastasis (LNM) in xenograft tumors of nude mice were observed.

**Results:**

The has-miR-506-3p was identified as the down-regulated gene in NPC based on the microarray data while LHX2 was negatively regulated by miR-506. Over-expression of miR-506 or silencing of LHK2 inhibited NPC cell proliferation, migration, invasion, tumorigenicity and LNM but promoted apoptosis indicated by decreased Wnt1, β-catenin, Vimentin, TCF4 and Twist expressions along with increased E-cadherin expressions.

**Conclusions:**

miR-506 inhibits tumor growth and metastasis in NPC via inhibition of Wnt/β-catenin signaling by down-regulating LHX2, accompanied by decreased TCF4. Taken together, miR-506 targeted-inhibition LHX2 presents a promising therapeutic strategy for the treatment of NPC.

**Trial registration:**

ChiCTR1800018889. Registered 15 October 2018.

**Electronic supplementary material:**

The online version of this article (10.1186/s13046-019-1023-4) contains supplementary material, which is available to authorized users.

RETRACTED

## Background

Nasopharyngeal carcinoma (NPC) is a tumor of the head and neck, derived from epithelial cells located in the nasopharynx, and is malignant in nature accompanied by early distant metastasis and local invasion, with a high incidence in southern China [1, 2]. Epstein-Barr virus infection, tumor suppressors, oncogenes and environmental factors are associated with the tumorigenesis of NPC, but the molecular mechanism of its pathogenesis remains to be completely clarified [3]. Though enhanced susceptibility to radiotherapy and excellent local control can be achieved with advances in radiotherapy and chemotherapy, the effectiveness of these treatments requires further improvements, especially with distant metastasis rates and high local recurrence rates [4]. In fact, 30% ~ 40% of NPC patients will develop distant metastasis within 4 years, and the prognoses become poor upon metastasis [5]. Metastasis, related to poor prognosis and death of cancer, is primarily responsible for the recurrence and initiating metastatic behaviours [6]. Moreover, the acquisition of metastatic potential in cancer cells including NPC cells, promotes the epithelial-mesenchymal transition (EMT), characterized by the loss of epithelial markers, the gain of mesenchymal markers as well as enhanced migration and invasion [7–9]. With a better understanding of the molecular mechanism controlling EMT process, targeting EMT multiple stages as a therapeutic target could benefit the treatment of epithelial malignancy and metastasis [10].

MicroRNAs (miRNAs) act as oncogenes or tumor suppressors owing to their role in the regulation of tumor metastasis, probably facilitating a new aspect to explore the underlying mechanisms in NPC progression [11, 12]. MiRNAs are short (~ 22 nucleotides) non-coding RNA molecules that can regulate gene expressions, while their dysfunction partially induces the development of cancer [13]. Strikingly, abnormal miRNA expressions have been observed in cases of NPC as well [14]. For instance, over-expression of miR-519 has been demonstrated to significantly suppress the development of NPC [15]. In addition, miR-506 has also been found to be down-regulated in NPC cell lines and tissues acting as a tumor suppressor via inhibition of the Forkhead box Q1, which is associated with tumor metastasis and proliferation in various cancers [16]. In the current study, we employed the website of microRNA.org, which predicated that miR-506 was able to target LHX2. LHX2, also known as LIM Homeobox 2, is up-regulated during EMT, followed by cell migration, invasion and metastatic dissemination [17]. Moreover, EMT has been previously related to high expression and nuclear accumulation of β-catenin [18, 19], indicating the possible involvement of the Wnt/β-catenin signalling pathway. Currently, only a few studies have explored the mechanism of cooperation of miR-506 and LHX2 in NPC. Therefore, we aimed to explore the effects of miR-506 in EMT and lymph node metastasis (LNM) in NPC via the Wnt/β-catenin signalling pathway by targeting LHX2, in the hope of providing a novel target for the treatment of NPC.

RETRACTED

## Materials and methods

### Ethics statement

The current study was approved by the Ethic Committee of the First Affiliated Hospital of Zhengzhou University. Signed informed consents were obtained from all patients.

### Microarray-based gene expression profiling

Based on the Gene expression Omnibus (GEO) database (http://www.ncbi.nlm.nih.gov/geo), chip data (GSE12425, GSE13597, GSE53819, and GSE64634) and annotation files related to “Nasopharyngeal carcinoma” were retrieved and downloaded. The included 4 chips data contained normal control samples and NPC samples. The two sample groups in each chip data were conducted with variance analysis using the Limma package of the R software. The differentially expressed genes were screened using *p* < 0.05 and |logFC| > 2 as the threshold. Next, heat maps based on the first 30 differentially expressed genes in each chip data were plotted using the pheatmap package of the R software, while Venn diagrams of the first 100 differentially expressed genes in each chip data by a Venn diagrams composition website (http://bioinformatics.psb.ugent.be/webtools/Venn/). Subsequently, the intersection of the four chips data was obtained.

### MiRNAs prediction

The miRNAs that could regulate LHX2 were retrieved from TargetScan (http://www.targetscan.org/vert_71/) (species: human), and then analytic results were enrolled from Conserved sites. In the DIANA (http://diana.imis.athena-innovation.gr/DianaTools/index.php?r=microT_CDS/index) (species: human) database, “LHX2” served as the key word, and a number of miRNAs were predicted in the database. For the purposes of improving the analysis accuracy, predicted miRNAs obtaining point > 0.9 were enrolled in the current study. Furthermore, miRDB (http://mirdb.org/miRDB/index.html), microRNA.org (http://34.236.212.39/microrna/home.do) and mirDIP (http://ophid.utoronto.ca/mirDIP/index.jsp#r; Minimum Score: Very High) were employed in order to predict miRNAs that could regulate LHX2. Prediction results from the above five datasets were analyzed based on Venn diagrams composition website, and the intersection was obtained.

### Study subjects

NPC tissues were collected from 78 patients who were diagnosed with primary NPC at the First Affiliated Hospital of Zhengzhou University, including 56 males and 22 females. The included patients were aged between 28 to 71 years, with the calculated mean age being 46.5 years. Based on the 2008 tumor node metastasis (TNM) staging system of NPC in China, the included tissues comprised of 5 cases of Stage I, 11 cases of Stage II, 46 cases of Stage III and 16 cases of Stage IV. Patients were enrolled into the current study if their first diagnosis was NPC; they did not undergo radiotherapy, chemotherapy or biotherapy prior to the surgery; they had no history of resection or metastatic disease; they did not suffer from other primary tumors [20]. All included patients had complete clinical data. After collection, the fresh tissues were frozen in liquid nitrogen for RNA isolation.

RETRACTED

### Hematoxylin-eosin (HE) staining

Tissue samples were fixed in 4% paraformaldehyde for over 24 h, dehydrated with 70% ethanol for 12 h, 80% ethanol for 6 h, 85% ethanol for 1 h, 90% ethanol for 1 h, 95% ethanol for 1 h, absolute ethyl alcohol for 30 min, 100% ethanol twice (each for 30 min), dewaxed in xylene for 2 h and in xylene II for 20 min, dehydrated and cleared. The tissue samples were sliced into 4 μm thick serial sections, attached onto slides in warm water, dried in a 38 °C oven overnight and then preserved at room temperature for further experimentation. The prepared section samples were dewaxed twice in xylene (approximately 10 min each time), dehydrated with 100, 95, 85 and 70% ethanol (each for 5 min), immersed in distilled water and stained with hematoxylin for about 10 min. After the removal of remaining dying solution by distilled water and addition of ethanol containing 0.5% ~ 1% hydrochloric acid for differentiation, the sections were observed under a microscope. When the nuclei and intra-nuclear chromosomes were clear, the sections were washed in water for 15 min, stained with 0.1% ~ 0.5% eosin for 1 min, washed in water for 1 min, dehydrated with 70, 80, 95 and 100% ethanol (each for 5 min), cleared, followed by the removal of additional liquid, and then mounted with neutral balsam and sealed. Histological changes were observed under an optical microscope.

### Reverse transcription-quantitative polymerase chain reaction (RT-qPCR)

Trizol (16,096,020, Thermo Fisher Scientific, Waltham, MA, USA) was employed to extract the total RNA content from tissues and cells. Total RNA (5 μg) was used as a template for reverse transcription reaction into cDNA following the instructions of a RT-qPCR kit (Applied Biosystems, Grand Island, NY, USA). The reaction amplification system was 25 μL, and the system were shown as follows: 300 ng cDNA, 1 × PCR buffer solution, 200 μmol/L dNTPs, 80 pmol/L PCR Forward Primer, 80 pmol/L PCR Reverse Primer, 0.5 U Taq enzyme (S10118, Shanghai Yuanye Biotech Co., Ltd., Shanghai, China). The reaction conditions were as follows: pre-degeneration at 94 °C for 5 min, and 30 cycles of denaturation at 94 °C for 30 s, annealing at 54.5 °C for 30 s, and extension at 72 °C for 30 s, followed by final extension at 72 °C for 10 min. The obtained product was preserved at 4 °C. Primers of miR-506, LHX2, Wnt1, β-catenin, E-cadherin, Vimentin, Twist, U6 and glyceraldehyde-3-phosphate dehydrogenase (GAPDH) were designed and synthesized by the TaKaRa Company (TaKaRa, Dalian, Liaoning, China) (Table 1). U6 was regarded as the internal reference for miR-506, while GAPDH for LHX2, Wnt1, β-catenin, E-cadherin, Vimentin and Twist. The 2^-ΔΔCt^ represented the ratio of the target genes in the experimental group to the control group, and the formula was as follow: ΔΔCT = ΔCt _experimental group_ - ΔCt _control group_, and ΔCt = Ct _target gene_ - Ct _internal reference_. Ct referred to the amplification cycle when the real-time fluorescence intensity of the reaction reached the set threshold and when the amplification was in the logarithmic growth. Each experiment was repeated three times to obtain the mean value.

RETRACTED

**Table 1:** Primer sequences for reverse transcription quantitative polymerase chain reaction

Gene	Forward (5′-3′)	Reverse (5′-3′)
miR-506	TAAGGCACCCTTCTGAGTAGA	GCGAGCACAGAATTAATACGAC
LHX2	CCGCCGCGATGCTGTTCCACAGTC	GAGTCATTAGAAAAGGTTGGTAAGAGTC
Wnt1	CCACCTCTTCGG CAAGA-TCGTCAA	GTGGCATTTGCACTCTTGGCGCAT
β-catenin	GCTGATTTGATGGAGTTGGA	TCAGCTACTTGTTCTTGAGTGAA
TCF4	CCCAGGACCCTGAGCTACTT	CTGGTGGCAACCCTGTAAGT
E-cadherin	GAGCCTGAGTCCTGCAGTCC	TGTATTGCTGCTTGGCCTCA
Vimentin	GAAGAGAACTTTGCCGTTGAAG	ACGAAGGTGACGAGCCATT
Twist	GTCCGCAGTCTTACGAGGAG	GCTTGAGGGTCTGAATCTTGCT
U6	TGACACGCAAATTCGTGAAGCGTTC	CCAGTCTCAGGGTCCGAGGTATTC
GAPDH	AGGTGAAGGTCGGAGTCAACG	GCTCCTGGAAGATGGTGATGG

Note: *miR-506* MicroRNA-506, *LHX2* LIM Homeobox 2, *TCF4* Transcription factor 4, *GAPDH* Glyceraldehyde-3-phosphate dehydrogenase

### Western blot analysis

Total protein content was extracted from 400 mg tissues using the Radio-Immunoprecipitation Assay (RIPA) lysate (Shanghai Shen Neng Bo Cai Biotechnology Co., Ltd., Shanghai, China). Next, the Bradford method was employed for total protein quantitation. The pre-treated protein was added to the sampling wells (each well about 20 μg) for protein isolation on 10% separation gel (120 V) and 5% spacer gel (60 V) for about 2 h. The protein samples were transferred onto the nitrocellulose membranes. A paper-gel-membrane-paper sandwich was set onto the electric transfer equipment, with gel at the negative electrode, nitrocellulose membrane at the positive electrode (voltage: 30 V; electrorotation: 12 h). After being blocked, the membranes were washed and incubated with rabbit monoclonal antibody against LHX2 (dilution ratio of 1: 2000, ab140614), rabbit polyclonal antibody against Wnt1 (dilution ratio of 1: 200, ab15251), rabbit monoclonal antibody against β-catenin (dilution ratio of 1: 5000, ab32572), rabbit monoclonal antibody against TCF4 (NCI-R159–6, dilution ratio of 1: 10000, ab217668), rabbit monoclonal antibody against E-cadherin (dilution ratio of 1: 10000, ab40772), rabbit monoclonal antibody against Vimentin (dilution ratio of 1: 2000, ab92547), rabbit polyclonal antibody against Twist (2.5 μg/mL, ab49254), rabbit polyclonal antibody cleaved caspase-3 (2.5 μg/mL, ab13585) and rabbit monoclonal antibody against GAPDH (dilution ratio of 1: 2500, ab9485) at 4 °C overnight. The membranes were washed and incubated with the secondary antibody of horse radish peroxidase (HRP)-labeled goat anti-rabbit immunoglobulin G (IgG) (dilution ratio of 1: 2000, ab6721) at 37 °C for 4 h. All aforementioned antibodies were purchased from Abcam Inc. (Cambridge, MA, USA). With the removal of Tris-buffered saline Tween-20 (TBST) using filter papers, the samples were placed on a clean glass plate. Equal amounts of A and B solutions of the enhanced chemiluminescence (ECL) kit (BB-3501, Ameshame, UK) were mixed avoiding exposure to light and added to the membranes for coloration. Densitometric analysis of the bands was carried out using the Gel imaging analysis system. Next, the Gel Doc XR imager system (Bio-Rad Laboratories, Inc., Hercules, CA, USA) was used for imaging and Quantity One (Bio-Rad version 4.6.2) for analysis. The gray value ratio of target protein to internal reference (GAPDH) was regarded as the relative protein expression. Experiments were repeated three times to obtain the mean value. The aforementioned procedures were also applicable for cell experimentation.

RETRACTED

### Dual-luciferase reporter gene assay

The binding site between miR-506 and LHX2 3′-untranslated region (3’-UTR) was analyzed using the microRNA website (microrna.org), and further tested by dual-luciferase reporter gene assay. The pMIR-reporter was introduced by virtue of the restriction enzyme sites, Spe I and Hind III. A complementary sequence of the mutation site of the seed sequence was designed based on the LHX2-wide-type (WT). Next, the target fragment was inserted into the pMIR-reporter plasmid using T4 DNA ligase after treatment with restriction endonuclease. The rightly sequenced luciferase reporter plasmids WT and mutant-type (MUT) were respectively co-transfected with miR-506 into HEK-293 T cells (CRL-1415, Shanghai Xinyu Biological Technology Co., Ltd., Shanghai, China). After 48-h transfection, the cells were collected, lysed and centrifuged for 3 ~ 5 min, followed by the collection of supernatant. Based on the manufacturer’s specification, the dual-luciferase reporter assay kit (RG005, Beyotime Institute of Biotechnology, Shanghai, China) was employed to dissolve the Renilla luciferase assay buffer and firefly luciferase assay agent. Renilla luciferase assay buffer (100 μL/sample) was added with substrate in proportion of 1: 100 in order to prepare a Renilla luciferase assay working solution. Each sample (20 ~ 100 μL) was added with 100 μL firefly luciferase assay agent (or 100 μL Renilla luciferase assay working solution), mixed by a pipette, followed by determination of relative luciferase activity (RLU). The cell lysate of reporter gene was regarded as the blank control, and Renilla luciferase as the internal control. RLU = RLU _firefly luciferase_ / RLU _Renilla luciferase_ [21].

### Cell line selection

A total of 5 NPC cell lines NE1 (human NPC cell line), CNE2 (poorly differentiated nasopharyngeal squamous cell carcinoma cell line), 5-8F (human highly metastatic NPC cell line), HONE-1 (human NPC cell line), 6-10B (human NPC cell line) were purchased from Cell bank in Shanghai Institute of Life Sciences, Chinese Academy of Sciences (Shanghai, China). Cell line authentication was carried out according to the suggestions from ATCC cell line authentication (Additional file 1: Table S1), and all aforementioned cell lines were detected as negative by short tandem repeat (STR) mycoplasma, bacteria, yeast and fungus. Next, the cell lines were cultured, and endogenous expression of LHX2 in NPC cells at the logarithmic phase of growth was determined by Western blot analysis as previously described. The cell line exhibiting the highest positive expression of LHX2 was selected for further experimentation.

### Cell treatment

The NPC cell lines CNE2 and 5-8F were selected and sub-cultured in an incubator with 5% CO_2_ and saturated humidity at 37 °C with Roswell Park Memorial Institute (RPMI) 1640 culture medium containing 10% fetal bovine serum (FBS), 100 U/mL penicillin, and 100 U/mL penicillin/streptomycin solution. The culture medium was replaced after 24 h, and passage was conducted after 72 h. The 3rd passage NPC cells at the logarithmic phase of growth were grouped into the blank group (blank control without any transfection), negative control group (NC, NPC cells transfected with NC plasmid), miR-506 mimic group (NPC cells transfected with miR-506 mimic), miR-506 inhibitor group (NPC cells transfected with miR-506 inhibitor), small interfering RNA against LHX2 group (siRNA-LHX2, NPC cells transfected with siRNA-LHX2) and miR-506 inhibitor + siRNA-LHX2 group (NPC cells transfected with miR-506 inhibitor and siRNA-LHX2). The above plasmids were synthetized by Shanghai Sangon Biological Engineering Technology & Services Co., Ltd. (Shanghai, China). The cells at the logarithmic phase of growth were seeded in a 6-well plate. When cell density reached 30% ~ 50%, the cells were transfected according to the instructions of Lipofectamine 2000 (Invitrogen, Carlsbad, California, USA). Serum-free Opti-MEM (250 μL, Gibco, Grand Island, NY, USA) was used to dilute 100 pmol miR-506 mimic, miR-506 inhibitor, siRNA-LHX2, miR-506 inhibitor + siRNA-LHX2 and NC with a final concentration of 50 nM, followed by mixing and incubation at room temperature for 5 min. Another 250 μL serum-free Opti-MEM was used to dilute 5 μL Lipofectamine 2000, mixed and incubated at room temperature for 5 min. The plasmid solution and Lipofectamine solution were mixed, incubated at room temperature for 20 min. The above two solutions were mixed and incubated at room temperature for 20 min and added in cell culture well. Following incubation at 37 °C with 5% CO_2_ for 6 ~ 8 h, the cells were further cultured in a complete medium for 24 ~ 48 h for the following experiment.

RETRACTED

### Chromatin immunoprecipitation (ChIP) assay

Upon reaching 70 ~ 80% confluence, the cells were added with 1% formaldehyde and fixed for 10 min at room temperature in order to make DNA and protein crosslink. After crosslinking, DNA and protein were randomly broken-down by ultrasound for a total of 15 times (10 s/time, interval of 10 s) to obtain DNA fragments of the appropriate size. Next, the samples were centrifuged at 4 °C at 30237×g, and the supernatant was collected into two tubes, which were then respectively incubated with the addition of NC rabbit monoclonal antibody against IgG (ab109489, dilution ratio of 1: 100, Abcam Inc., Cambridge, MA, USA) and target protein specific mouse antibody against LHX2 (C-20, sc-19,344, Santa Cruz, Santa Cruz, CA, USA) overnight at 4 °C. Next, the endogenous DNA-protein complex was precipitated using Protein Agarose/Sepharose, centrifuged transiently and the supernatant was discarded. After the non-specific complex was washed, the crosslink was reversed overnight at 65 °C. DNA fragments were purified and recovered by phenol-chloroform extraction, and the primer of transcription factor 4 (TCF4) promoter fragment (forward sequence of 5’-TACAGCTCATAAAGGCAGTGTGGCC-3′ and reverse sequence of 5’-GGCGCTTGAGAAGCCCTTCAGCCCGC-3′) was used for RT-qPCR analysis [22].

RETRACTED

### Dual-luciferase reporter gene assay

The promoter region of TCF4 (grch38:18:55221731–55,665,387) was amplified using the following primer: 5’-TACAGCTCATAAAGGCAGTGTGGCC-3′ (forward) and 5’-GGCGCTTGAGAAGCCCTTCAGCCCGC-3′ (reverse). Next, the amplified fragments were purified and inserted into luciferase vector pGL3-Basic in order to construct the TCF4 reporter gene plasmid pGL3-Basic-TCF4 promotor. The cDNA of human LHX2 was sub-cloned into pCMV-SPORT6 vector to construct LHX2 expression plasmid pCMV-Lhx2. Thereafter, the TCF4 reporter gene and LHX2 expression plasmids were co-transfected into human embryonic kidney HEK293T cells (purchased from the Cell Bank of the Typical Culture Preservation Committee of the Chinese Academy of Sciences). After 48-h transfection, the cells were collected and lysed. A luciferase detection kit (K801–200, Biovision Mountain View, CA, USA) and dual-luciferase reporter gene analysis system (Promega, Madison, WI, USA) were employed to detect the luciferase reporter gene. Renilla luciferase was regarded as the internal control and the luciferase activity of reporter gene was calculated as follows: RLU firefly luciferase / RLU Renilla luciferase × 100%.

### 3-(4,5-dimethyl-2-thiazolyl)-2,5-diphenyl-2-H-tetrazolium bromide (MTT) assay

After transfection, the cells were allowed to grow with adherence for 24 h. When cell density reached about 80%, the cell samples were rinsed with phosphate buffer saline (PBS) twice, and detached with 0.25% trypsin in order to prepare a single cell suspension. A total of 6 wells with treated cells and fresh RPMI 1640 culture medium were reacted with 10% MTT solution (5 g/L, GD-Y1317, Guduo Biotechnology Company, Shanghai, China) at 37 °C for 4 h. Following the formation of water-insoluble blue violet formazan crystals, the medium was discarded. Next, the cells were rinsed with PBS twice, added with 150 μL dimethyl sulfoxide (DMSO, D5879-100ML, Sigma-Aldrich, St. Louis, MO, USA) and shaken for 5 min. Subsequently, the optical density (OD) values of each well were measured using an excitation wavelength of 570 nm by a microplate reader (Nanjing DeTech Experimental Equipment Co., Ltd., Nanjing, Jiangsu, China). The experiment was repeated three times to obtain the mean value. The time point was regarded as the abscissa, the OD value as the ordinate, and the cell viability curve was plotted.

### Flow cytometry

After 48-h transfection, the cells were collected, treated with serum-free medium for 48 h to synchronize the cell cycle, rinsed thrice with cold PBS, followed by centrifugation with the supernatant removed. Afterwards, the cells were resuspended with PBS and adjusted to a density 1 × 10^5^ cells/mL. Next, the cells were fixed in 1 mL pre-cooled (− 20 °C) 75% ethanol at 4 °C for 1 h, centrifuged with the removal of ethanol, and rinsed twice with PBS. After the supernatant was discarded, 100 μL RNaseA (GE101–01, TransGen Biotech Co., Ltd., Beijing, China) was added to the cells. Then the cells were placed under dark conditions at 37 °C in a water bath for 30 min, and stained with 400 μL propidium iodide (PI, 88378, Sigma-Aldrich, St. Louis, MO, USA) at 4 °C avoiding exposure to light for 30 min. Subsequently, the cell cycle was analyzed by detecting red fluorescence at the wavelength of 488 nm using a flow cytometer (CytoFLEX, Beckman Coulter, CA, USA).

RETRACTED

Annexin V-fluorescein isothiocyanate (FITC)/PI double staining was performed to detect the cell apoptosis 48 h after transfection. The cells were detached by ethylenediaminetetraacetic acid (EDTA)-free 0.25% trypsin (YB15050057, Shanghai Bo Yu Biological Technology Co., Ltd., Shanghai, China), collected into a flow tube, and centrifuged with the supernatant removed, followed by 3 cold PBS rinses. Following centrifugation, the supernatant was discarded. Based on the instructions of the Annexin V-FITC/PI Apoptosis Detection kit (K201–100, BioVision, Milpitas, CA, USA), Annexin-V-FITC/PI dye was prepared using Annexin-V-FITC, PI, hydroxyethyl piperazine ethanesulfonic acid (HEPES) using a 1: 2: 50 ratio. Every 100 μL of dye liquor was used to re-suspend 1 × 10^6^ cells, followed by oscillation and mixing. The specimens were then cultured at room temperature for 15 min, followed by the addition of 1 mL HEPES buffer (PB180325, Procell Life Science & Technology Co., Ltd., Wuhan, Hubei, China), oscillation and mixing accordingly. Cell apoptosis was analyzed through the detection of FITC and PI fluorescence by activating the band pass at 515 nm and 620 nm by a wavelength of 488 nm using flow cytometer. Experiments were repeated three times to obtain the mean value.

### Scratch test

Cells in good conditions at the logarithmic phase of growth were seeded in a 6-well plate (cell density of 1 × 10^6^ cells/well) and cultured in a 5% CO_2_ incubator at 37 °C. The following day, when cell density reached 80% ~ 90%, the medium was replaced with a serum-free medium for 24-h cell starvation. A wound was created using a sterile 200-μL pipette straight along the scratch line. Next, the cells were rinsed with sterile PBS to remove the debris. Each well was added with serum-free medium and incubated in a 5% CO_2_ incubator at 37 °C with saturated humidity. Images of the wounds were acquired for measurement of scratch width (migration distance) as an indicator of wound healing at 0 h and 24 h under an inverted microscope. Experiments were repeated three times to obtain the mean value.

RETRACTED

### Transwell assay

The prepared Matrigel was dissolved in the apical chamber of an incubator. Each chamber was added with 2 drops of serum-free medium for modifying hydrophilic materials on the membrane and cultured in an incubator. Next, the basal chamber with 500 μL full serum medium was added into the chamber. After 24-h transfection, the cells were detached by trypsin, centrifuged, collected, rinsed with PBS twice, and re-suspended in serum-free Dulbecco’s modified Eagle’s medium (DMEM) to a density of 5 × 10^4^ cells/200 μL. The basolateral chamber was added with a RPMI 1640 medium containing 10% FBS as chemotactic factor, and the apical chamber with 200 μL cell suspension. After being cultured for 24 h, the cells that did not move through the Matrigel on the apical chamber were removed using cotton slivers. The Transwell chambers were fixed with 70% ethanol for 15 min, washed 3 times with PBS, air-dried, stained with hematoxylin for 15 min and rinsed 3 times with double distilled water. The chamber was dried at room temperature, cut off using blade, placed on a slide with a drop of xylene, cleared for 2 ~ 5 min, mounted with neutral balsam, sealed and observed. A minimum of 5 fields of vision were randomly selected from each sample to calculate the mean number of cells that had moved through the Matrigel as the index of cell invasion ability.

### Xenograft tumors in nude mice

BALB/c-nu male nude mice (age: 3 ~ 5 weeks; weight: 20 ~ 28 g) (Experimental Animal Center of Guangxi Medical University, Nanning, Guangxi, China) were grouped into blank, NC, miR-506 mimic, miR-506 inhibitor, siRNA-LHX2 and miR-506 inhibitor + siRNA-LHX2 groups, with at least 12 mice in each group. CNE2 cell line at the logarithmic phase of growth was labeled by green fluorescence, and then detached by trypsin and counted. The nude mice were subcutaneously injected with 0.2 mL cell suspension (1.0 × 10^7^ cells/mL) in the foot-pads. The maximum diameter (a) and minimum diameter (b) of tumor that appeared in mice were measured once every 2 d using Vernier calipers to calculate the tumor volume according to the formula as follows: Volume = (a × b)/2. Additionally, volume change and LNM of xenograft tumor were observed by a small-animal imaging system (Lumozone FA1024, MAG Biosystems analysis software, Experimental Animal Center of Guangxi Medical University, Nanning, Guangxi, China) for consecutive 28 d [23, 24]. The nude mice were anaesthetized via intraperitoneal injection of 1% pentobarbital sodium, and placed in a dosal position on a glue pad of animal living imaging system. Tumor fluorescence absorption value was detected at different time intervals, d_4_, d_8_, d_12_, and d_16_ (Irradiation condition: Green Fluorescent Protein (GFP), Emission wavelength: 520 nm, Excitation wavelength: 480 nm, Exposure time: 5 ms). Subsequently, the number of tumor-bearing mice that suffered from LNM and the number of LNM (armpit and groin) were counted. Next, the lymph node and the xenograft tumors (primary tumors) were isolated, fixed in 10% formalin, embedded with paraffin, sectioned, stained with hematoxylin and eosin and observed under a light microscope. Then, cell proliferation and apoptosis in partial tumor tissues were detected by Immunohistochemistry using antibodies against cleaved Caspase-3 (ab32351) and Ki67 (ab15580) purchased from Abcam Inc. (Cambridge, MA, USA). The remaining tumor tissues were used for RT-qPCR and Western blot analysis.

RETRACTED

### Statistical analysis

Statistical analyses were performed using the SPSS 21.0 software (IBM Corp., Armonk, NY, USA). Measurement data was presented as mean ± standard deviation. Normal distribution and skewed distribution tests were performed for all included data. Comparisons between two groups were performed using the *t*-test, and non-parametric tests (i.e. Mann-Whitney U test) were applied for data with highly skewed distribution. Comparisons among multiple groups were assessed by one-way analysis of variance (ANOVA), and non-parametric tests (i.e. Kruskal-Wallis H test) were applied for data with highly skewed distribution. Enumeration data were expressed as ratio or percentage and analyzed by the *chi*-square tests. A value of *p* < 0.05 was considered to be statistically significant.

## Results

### miR-506-3p and LHX2 are involved in NPC

A total of 4 NPC-related chip data, namely, GSE12425, GSE13597, GSE53819 and GSE64634 were screened using the GEO database for the identification of differentially expressed genes. There were 766 differentially expressed genes in GSE12425, 602 in GSE13597, 478 in GSE53819, and 1032 in GSE64634, amounting to a total of 2878 genes. Heat maps based on the first 30 differentially expressed genes in each chip data were plotted, as shown in Fig. 1a-d. Venn diagrams of the first 100 differentially expressed genes in each chip data were drawn, and the intersection was obtained (Fig. 1e). The results indicated that solely the LHX2 gene was found at the intersection, with its high expression in NPC recorded in the four datasets. Based on the aforementioned findings, we hypothesized that LHX2 may promote the progression of NPC. Further research revealed that existing literature had reported that the Wnt/β-catenin signaling pathway was closely related to the progression of NPC [25–28]. Moreover, a few studies have documented that LHX2 mediates the Wnt/β-catenin signaling pathway in the development of disease [29, 30]. However, the mechanism by which LHX2 affects NPC remains to be unclear. Additionally, the effect of LHX2 on the Wnt/β-catenin signaling pathway in NPC needs further clarification. To further understand the mechanism of LHX2 in NPC, we employed a miRNA dataset to predict miRNAs that could regulate LHX2. In the current study, 5 different databases were employed to improve the accuracy of the prediction results. In TargetScan database, 14 predicted miRNAs from Conserved sites were assessed in subsequent analyses. In DIANA database, 35 miRNAs getting point > 0.9 from 154 predicted miRNAs were enrolled in the current study. A total of 54, 23 and 35 nonredundant miRNAs predicted from miRDB, microRNA.org and mirDIP database, respectively. Venn diagrams of the above 5 datasets were drawn, and the intersection was obtained (Fig. 1f). The intersection revealed that has-miR-506-3p was related to the expression of LHX2. The findings above signified that has-miR-506-3p might regulate LHX2 expression and mediate the Wnt/β-catenin signaling pathway in NPC.

RETRACTED

**Fig. 1:** has-miR-506-3p regulated LHX2 expression and mediated the Wnt/β-catenin signaling pathway in NPC by microarray profiling. **a**-**d** heat maps with hierarchical clustering analysis on the microarray dataset GSE12425, GSE13597, GSE53819 and GSE64634 show differentially expressed genes. The abscissa represents the sample number, while the ordinate shows the gene name. The histogram of the upper right is a color order. The color change from top to bottom indicates that the expression of sample is from high to low. Each rectangle corresponds to the expression of sample, and each column represents the expression of all genes in each sample. The left dendrogram indicates the result of cluster analysis of different genes from different samples. The top bar represents the sample type, and the upper right box represents the color of the sample. The blue is the normal control sample, and the red is the tumor sample. **e** Venn diagrams of dataset GSE12425 (blue), GSE13597 (red), GSE53819 (green) and GSE64634 (yellow) show the number of differentially expressed genes. The middle part as the blue arrow shown represents the intersection of four datasets. **f** Venn diagrams of predicted miRNAs from the databases of TargetScan (blue), DIANA (red), miRDB (brown), microRNA.org (yellow) and mirDIP (green). The middle part as the blue arrow shown represents the intersection of f datasets

### miR-506 is down-regulated while LHX2 is up-regulated in NPC tissues

We employed RT-qPCR and Western blot analysis in order to determine the expressions of miR-506, LHX2, Wnt1, β-catenin, E-cadherin, Vimentin, and Twist in the NPC and paracancerous tissues. The expressions of miR-506 and mRNA levels of E-cadherin were found to be decreased in NPC tissues in comparison to those in paracancerous tissues, but the mRNA levels of LHX2, Wnt1, β-catenin, Vimentin, and Twist were elevated (all *p* < 0.05) (Fig. 2a). When compared with paracancerous tissues, the NPC tissues showed a decrease in the protein levels of E-cadherin and an increase in the protein levels of LHX2, Wnt1, β-catenin, Vimentin, and Twist (all *p* < 0.05) (Fig. 2b and c). These results proved that miR-506 was poorly expressed while LHX2 was highly expressed in NPC tissues.

RETRACTED

**Fig. 2:** miR-506 was down-regulated while LHX2 was up-regulated in NPC tissues. **a** the miR-506 expression and mRNA level of LHX2, Wnt1, β-catenin, E-cadherin, Vimentin, and Twist in NPC and paracanerous tissues as determined by RT-qPCR; **b** and **c** the protein level of LHX2, Wnt1, β-catenin, E-cadherin, Vimentin, and Twist in NPC and paracanerous tissues as measured by western blot analysis; * *p* < 0.05 vs. the paracancerous tissue; miR-506, microRNA-506; LHX2, LIM Homeobox 2; E-cadherin, epithelial-cadherin; NPC, nasopharyngeal carcinoma; RT-qPCR, reverse transcription-quantitative polymerase chain reaction

### LHX2 is a target gene of miR-506

Furthermore, we examined whether miR-506 could directly regulate LHX2 by means of target prediction program and luciferase activity determination. The microRNA.org website predicated that miR-506 was able to target LHX2 as a result of the existence of specific binding sites between LHX3 3’UTR and miR-506. In order to verify that LHX2 was a direct target gene of miR-506, the dual-luciferase reporter gene assay was applied and the results displayed that compared with the NC group, the luciferase activity of wild-type LHX2 3’-UTR was inhibited by miR-506 (*p* < 0.05), while that of mutant 3’-UTR didn’t exhibit the same effect (*p* > 0.05) (Fig. 3). These findings indicated that miR-506 may specifically bind to LHX2–3’-UTR and down-regulate LHX2 gene expression at a post-transcriptional level. The aforementioned results suggested that miR-506 might directly target LHX2.

**Fig. 3:** LHX2 was a target gene of miR-506. **a** the predicted relationship between miR-506 and LHX2 by bioinformatics prediction website; **b** the targeting relationship between miR-506 and LHX2 verified by dual-luciferase reporter gene assay; * *p* < 0.05 vs. the NC group; NC, negative control; miR-506, microRNA-506; LHX2, LIM Homeobox 2

RETRACTED

### CNE2 and high metastatic 5-8F cell lines present with the highest LHX2 expression

Western blot analysis was further performed to select the qualified cell line for subsequent experiments in terms of the LHX2 expression. The protein expressions of LHX2 were found to be higher in the CNE2 cell line in comparison with the CNE1, 5-8F, HONE-1 and 6-10B cell lines (Fig. 4). Therefore, CNE2 and high metastatic 5-8F cell lines with the highest LHX2 expression were selected for the further experimentation.

**Fig. 4:** The highest LHX2 expression was found in CNE2 and high metastatic 5-8F cell lines. **a** the expression pattern of LHX2 in NPC cell lines as determined by Western blot analysis; **b** the histogram of LHX2 expression in NPC cell lines; * *p* < 0.05 vs. the CNE2 cell line; LHX2, LIM Homeobox 2

### MiR-506 inactivates the Wnt/β-catenin signaling pathway in NPC cells

A previous study revealed that LHX2 can directly target and regulate TCF4 [22]. In addition, LHX2 was reported to be capable of disrupting the Wnt/β-catenin signaling pathway, and furthermore that the signaling pathway can bind with TCF4 to regulate tumor cell growth and apoptosis [31, 32]. RT-qPCR and Western blot analysis were employed to determine the relative mRNA and protein levels of related genes in CNE2 cell lines following transfection. Compared with the blank and NC groups, the miR-506 mimic and siRNA-LHX2 groups showed elevated miR-506 expressions as well as mRNA and protein levels of E-cadherin, and decreased mRNA and protein levels of LHX2, Wnt1, β-catenin, TCF4, Vimentin, and Twist (all *p* < 0.05); the miR-506 inhibitor group presented with reduced miR-506 expressions and mRNA and protein levels of E-cadherin, in addition to increased mRNA and protein levels of LHX2, Wnt1, β-catenin, TCF4, Vimentin, and Twist (all *p* < 0.05); the miR-506 inhibitor + siRNA-LHX2 group revealed exhibited expressions of miR-506 (*p* < 0.05). No differences regarding the mRNA and protein levels of E-cadherin, LHX2, Wnt1, β-catenin, TCF4, Vimentin, and Twist were observed among the blank, NC and miR-506 inhibitor + siRNA-LHX2 groups (all *p* > 0.05, Fig. 5a, b, g and h).

**Fig. 5:** miR-506 suppressed the Wnt/β-catenin signaling pathway in NPC cells by inhibiting LHX2. **a** the miR-506 expression and mRNA level of LHX2, Wnt1, β-catenin, E-cadherin, Vimentin, and Twist in CNE2 cells following transfection as determined by RT-qPCR; **b** the protein level of LHX2, Wnt1, β-catenin, E-cadherin, Vimentin, and Twist in CNE2 cells following transfection as measured by Western blot analysis; **c** the miR-506 expression and mRNA level of LHX2, Wnt1, β-catenin, E-cadherin, Vimentin, and Twist in 5-8F cells following transfection as determined by RT-qPCR; **d** protein bands and the protein level of LHX2, Wnt1, β-catenin, E-cadherin, Vimentin, and Twist in 5-8F cells following transfection as measured by Western blot analysis; **e** the binding of LHX2 and IgG with the promoter region of TCF4 in CNE2 and 5-8F cells as determined by ChIP assay; **f** the binding of LHX2 with the promoter of TCF4 as determined by dual-luciferase reporter gene assay; **g** and **i** mRNA level of TCF4 in CNE2 and 5-8F cells following transfection as determined by RT-qPCR; **h** and **j** protein bands and the protein level of TCF4 in CNE2 and 5-8F cells following transfection as measured by Western blot analysis; * *p* < 0.05, vs. the blank and NC groups; NC, negative control; miR-506, microRNA-506; LHX2, LIM Homeobox 2; NPC, nasopharyngeal carcinoma; E-cadherin, epithelial-cadherin; RT-qPCR, reverse transcription-quantitative polymerase chain reaction; TCF4, transcription factor 4; IgG, immunoglobulin G

Next, results of ChIP and dual-luciferase reporter gene assay displayed that LHX2 can bind to the promoter region of TCF4, and enhance the activity of TCF4 promoter (Fig. 5e and f). Detection of the expressions of miR-506, LHX2, Wnt1, β-catenin, E-cadherin, TCF4, Vimentin, and Twist in 5-8F cell lines after transfection was ensued, and the results were similar to those of the CNE2 cell lines (Fig. 5c, d, i and j).

RETRACTED

These results suggested that restored miR-506 inhibited LHX2 expression, which reduced TCF4 expression and then inactivated the Wnt/β-catenin signaling pathway, therefore suppressing the expression of EMT-related factors indicated through up-regulation of E-cadherin and repression of Vimentin.

### Up-regulation of miR-506 or silencing LHX2 inhibits NPC cell proliferation

MTT assay was performed in order to assess the effects of miR-506 on cell vitality in all groups. Relative vitality of CNE2 and 5-8F cells following transfection in each group is shown in Fig. 6. No differences regarding cell vitality at the 24-h time point were found among the groups (*p* > 0.05). In contrast to the blank and NC groups after 24-h transfection, the miR-506 mimic and siRNA-LHX2 groups exhibited inhibited cell vitality, while the miR-506 inhibitor group showed enhanced cell vitality at 48 h and 72 h (all *p* < 0.05). Cell vitality did not differ significantly among the blank, NC and miR-506 inhibitor + siRNA-LHX2 groups (*p* > 0.05). Similarly, there were no differences regarding cell vitality between the miR-506 mimic and siRNA-LHX2 groups (*p* > 0.05). All results above indicated that the proliferation of CNE2 cells decreased following transfection with miR-506 mimic or siRNA-LHX2.

RETRACTED

**Fig. 6:** Up-regulation of miR-506 or silencing of LHX2 repressed NPC cell proliferation. **a** the cell viability curves of CNE2 cells following transfection as measured by MTT assay; **b** the cell viability curves of 5-8F cells following transfection as assessed by MTT assay; * *p* < 0.05, vs. the blank and NC groups; MTT, 3-[4,5-dimethylthiazol-2-yl]-2,5-diphenyl tetrazolium bromide; NC, negative control; miR-506, microRNA-506; NPC, nasopharyngeal carcinoma; LHX2, LIM Homeobox 2

### Up-regulation of miR-506 or silencing LHX2 affects NPC cell cycle

Flow cytometry was performed in order to investigate miR-506 and LHK2 and their respective effects on cell cycle of NPC cells. The results of PI single staining are shown in Fig. 7a. The miR-506 mimic and siRNA-LHX2 groups showed more cells in the G1 phase and fewer cells in the S phase in comparison with the blank and NC groups, but the miR-506 inhibitor exhibited opposite trends (all *p* < 0.05). No differences concerning the number of cells in the G1, S and G2 phase were observed among the blank, NC and miR-506 inhibitor + siRNA-LHX2 groups (all *p* > 0.05). Similarly, there were no differences in the number of cells in the G1, S and G2 phase between the miR-506 mimic and siRNA-LHX2 groups (all *p* > 0.05). However, the number of cells in the G2 phase was found to be not obviously different among the six groups (all *p* > 0.05). The same results were obtained from the 5-8F NPC cell line following transfection (Fig. 7b). These findings demonstrated that up-regulated miR-506 or down-regulated LHX2 increased the proportion of cells in the G1 phase and reduced that of cells in the S phase, signifying that up-regulating miR-506 or silencing LHX2 might be responsible for changes in NPC cell cycle.

**Fig. 7:** Up-regulation of miR-506 or silencing of LHX2 influenced NPC cell cycle. **a** the DNA content of PI-stained CNE2 cells at the G0/G1, S, and G2/M phases as assessed by flow cytometry; **b** the DNA content of PI-stained 5-8F cells at the G0/G1, S, and G2/M phases as evaluated by flow cytometry; * *p* < 0.05, vs. the blank and NC groups; NC, negative control; miR-506, microRNA-506; NPC, nasopharyngeal carcinoma; LHX2, LIM Homeobox 2; PI, propidium iodide

### Up-regulation of miR-506 or silencing LHX2 promotes NPC cell apoptosis

Flow cytometry analyses of Annexin-V/PI double staining were performed in order to investigate the effect of miR-506 and LHX2 on cell apoptosis of NPC cells as shown in Fig. 8a. In comparison with the blank and NC groups, cell apoptosis was found to be promoted in the miR-506 mimic and siRNA-LHX2 groups, while inhibited in the miR-506 inhibitor group (all *p* < 0.05). There were no significant cell apoptosis differences among the blank, NC and miR-506 inhibitor + siRNA-LHX2 groups (*p* > 0.05). Similarly, there were no differences in cell apoptosis between the miR-506 mimic and siRNA-LHX2 groups (*p* > 0.05). Additionally, Western blot analysis was employed to determine the expression pattern of cleaved Caspase 3 in the NPC cell line following transfection so as to further confirm the effect of miR-506 and LHX2 on cell apoptosis (Fig. 8c). The results suggested that in comparison with the blank and NC groups, the protein levels of cleaved Caspase-3 were increased in the miR-506 mimic and siRNA-LHX2 groups, while decreased levels were observed in the miR-506 inhibitor group (*p* < 0.05); however, no significant differences regarding the protein levels of cleaved caspase-3 were observed in the miR-506 inhibitor + siRNA-LHX2 group (*p* > 0.05). Likewise, identical results were obtained from the 5-8F NPC cell line following transfection as presented in Fig. 8b and d. All in all, the aforementioned results suggested that the up-regulation of miR-506 or silencing of LHX2 could promote the NPC cell apoptosis by regulating apoptosis-related signaling.

RETRACTED

**Fig. 8:** Up-regulation of miR-506 or silencing of LHX2 promoted NPC cell apoptosis. **a** the CNE2 cell apoptosis following transfection as determined by flow cytometry Annexin V/PI double parameter method; **b** the 5-8F cell apoptosis following transfection as evaluated by flow cytometry Annexin V/PI double parameter method; **c** the protein level of cleaved caspase-3 in CNE2 cells following transfection as determined by western blot analysis; **d** the protein level of cleaved caspase-3 in 5-8F cells following transfection as measured by western blot analysis; * *p* < 0.05, vs. the blank and NC groups; NC, negative control; miR-506, microRNA-506; NPC, nasopharyngeal carcinoma; PI, propidium iodide; LHX2, LIM Homeobox 2

### Up-regulation of miR-506 or silencing of LHX2 inhibits NPC cell migration

Furthermore, the current study performed a series of scratch tests to evaluate the effects of miR-506 and LHX2 on NPC cell migration. As shown in Fig. 9, in contrast with the blank and NC groups following 24-h transfection, the cell migration distance was found to be shortened in the miR-506 mimic and siRNA-LHX2 groups, while lengthened distances were observed in the miR-506 inhibitor group (all *p* < 0.05). No differences regarding cell migration abilities were observed among the blank, NC and miR-506 inhibitor + siRNA-LHX2 groups (*p* > 0.05). Similarly, there were no differences in cell migration between the miR-506 mimic and siRNA-LHX2 groups (*p* > 0.05). Correspondingly, same results were obtained from the 5-8F NPC cell line following transfection as shown in Fig. 9b. All results above suggested that NPC cell migration was decreased following transfection with miR-506 mimic or siRNA-LHX2.

RETRACTED

**Fig. 9:** Up-regulation of miR-506 or silencing of LHX2 hindered NPC cell migration. **a** CNE2 cell migration following transfection as measured by scratch test; **b** 5-8F cell migration following transfection as evaluated by scratch test; * *p* < 0.05, vs. the blank and NC groups NC, negative control; miR-506, microRNA-506; LHX2, LIM Homeobox 2; NPC, nasopharyngeal carcinoma

### Up-regulation of miR-506 or silencing LHX2 inhibits NPC cell invasion

The current study employed Transwell assay in order to assess the effects of miR-506 on CNE2 cell invasion following 24-h transfection (Fig. 10a). Compared with the blank and NC groups, the cell invasion ability was found to be weakened in the miR-506 mimic and siRNA-LHX2 groups, while enhanced in the miR-506 inhibitor group (all *p* < 0.05); no differences regarding cell invasion abilities were observed among the blank, NC and miR-506 inhibitor + siRNA-LHX2 groups as well as between the miR-506 mimic and siRNA-LHX2 groups (all *p* > 0.05); as expected, the aforementioned results were similar to the results obtained from the 5-8F NPC cell line following transfection as depicted in Fig. 10b. The aforementioned results proved that up-regulation of miR-506 or down-regulation of LHX2 inhibited the invasion of NPC cells.

**Fig. 10:** Up-regulation of miR-506 or silencing LHX2 suppressed NPC cell invasion. **a** CNE2 cell invasion following transfection as measured by Transwell assay; **b** 5-8F cell invasion following transfection as assessed by Transwell assay; * *p* < 0.05, vs. the blank and NC groups; NC, negative control; miR-506, microRNA-506; NPC, nasopharyngeal carcinoma; LHX2, LIM Homeobox 2

### Up-regulation of miR-506 or silencing LHX2 suppresses LNM and tumorigenicity in nude mice with NPC

The tumor xenograft procedure in nude mice was conducted in order to measure LNM and cell tumorigenicity, the results of which demonstrated that nude mice showed palpable tumor mass after 1 week of tumor bearing. The numbers of tumor bearing mice and LNM are shown in Fig. 11a-c. Four weeks after inoculation, in contrast to the blank and NC groups, the miR-506 mimic and siRNA-LHX2 groups exhibited reduced number of tumor bearing mice and LNM, whereas the miR-506 inhibitor group presented with opposite trends (*p* < 0.05). No differences regarding the number of tumor bearing mice, and LNMs were observed among the blank, NC and miR-506 inhibitor + siRNA-LHX2 groups (*p* > 0.05). Additionally, tumor volumes were calculated with the curve plotted (Fig. 11e). Compared with the blank and NC groups, tumor volume was found to be exhibit reduction from the 8th to the 14th d in the miR-506 mimic and siRNA-LHX2 groups, but increased from the 4th to the 14th d in the miR-506 inhibitor group (all *p* < 0.05); no obvious changes regarding tumor volume were detected in the miR-506 inhibitor + siRNA-LHX2 groups (*p* > 0.05). Fluorescence absorption of subcutaneous tumor in nude mice was determined using an animal-imaging instrument at various time intervals (4 d, 8 d, 12 d and 16 d). When compared to the blank and NC groups, the fluorescence absorption value was found to be decreased from the 8th d to the 16th d in the miR-506 mimic and siRNA-LHX2 groups but increased in the miR-506 inhibitor group (*p* < 0.05) (Fig. 11d). However, the miR-506 inhibitor + siRNA-LHX2 group exhibited no significant differences upon comparison with the blank and NC groups (*p* > 0.05). In addition, xenograft tumor tissues were stained with hematoxylin and eosin and observed under a light microscope (Fig. 11f). It was found that the xenograft tumor tissues from each group were wrapped with fibrous connective tissues with obvious interstitial edema. Compared with the blank and NC groups, keratinocyte carcinoma, tumor necrosis area, more nuclear fission and obvious lymphocyte infiltration were observed in the miR-506 mimic and siRNA-LHX2 groups, whereas the miR-506 inhibitor group showed less neoplasm necrosis, nuclear fission and lymphocyte infiltration. The results were not significantly different in the miR-506 inhibitor + siRNA-LHX2 group whom compared to the blank and NC groups (*p* > 0.05).

RETRACTED

**Fig. 11:** Up-regulation of miR-506 or silencing LHX2 suppressed LNM, and tumorigenicity in nude mice with NPC. **a** images of the lymph node metastatic sites in nude mice following intraperitoneal injection; **b** the number of tumor-bearing mice with LNM following intraperitoneal injection; **c** the number of LNM; **d** the fluorescence absorption value of tumor in each group; **e** tumor growth curves in each group; **f** pathological changes of xenograft tumor tissues detected by HE staining; * *p* < 0.05, vs. the blank and NC groups; LNM, lymph node metastasis; NC, negative control; miR-506, microRNA-506; NPC, nasopharyngeal carcinoma; LHX2, LIM Homeobox 2; E-cadherin, epithelial-cadherin; HE, hematoxylin-eosin; RT-qPCR, reverse transcription-quantitative polymerase chain reaction

These findings demonstrated that up-regulated miR-506 or down-regulated LHX2 delayed the growth of xenograft tumors, ameliorated NPC and suppressed LNM.

### Up-regulation of miR-506 or silencing LHX2 hinders tumor growth in NPC

To further elucidate the effects of miR-506 on the tumor growth, the expression pattern of Ki67 and cleaved caspase-3 in xenograft tumor tissues of mice was measured using Immunohistochemistry. As shown in Fig. 12a and b, compared with the blank and NC groups, the number of Ki67 positive cells was found to be significantly decreased in the miR-506 mimic and siRNA-LHX2 groups, while the number of cleaved caspase-3 positive cells was notably increased; an opposite trend was observed in the miR-506 inhibitor group. Furthermore, the results of determination of miR-506 expression by RT-qPCR as well as measurement of LHX2, Wnt1, β-catenin, E-cadherin, Vimentin, and Twist protein levels by Western blot analysis in tumor tissues demonstrated consistent results with in vitro intervention (Fig. 12c and d). Altogether, over-expressed miR-506 or silenced LHX2 inhibited the tumor growth.

RETRACTED

**Fig. 12:** Up-regulation of miR-506 or silencing LHX2 inhibited tumor growth. **a** the positive expression rate of Ki67 protein in xenograft tumor tissues as measured by Immunohistochemistry; **b** the positive expression rate of Caspase-3 protein in xenograft tumor tissues as assessed by Immunohistochemistry; **c** miR-506 expression in xenograft tumor tissues as determined by RT-qPCR; **d** the protein levels of LHX2, Wnt1, β-catenin, E-cadherin, Vimentin, and Twist in xenograft tumor tissues as measured by western blot analysis; miR-506, microRNA-506; LHX2, LIM Homeobox 2; EMT, epithelial mesenchymal transition; NC, negative control; RT-qPCR, reverse transcription-quantitative polymerase chain reaction

## Discussion

NPC is a malignant tumor owing to its highly invasive and metastatic potential [33]. Metastasis, a primary hallmark of malignant tumors, is responsible for most cancer-related deaths [34]. Multimodal treatment for the local control of NPC has achieved great advances with better improvement; however, distant metastasis is still regarded as the most frequent failure pattern [35]. Therefore, better understanding of the molecular patterns of NPC metastasis is crucial in order to develop novel treatment strategies effective to patients with NPC. In NPC cases, dysregulated miRNA expressions have been observed, and the abnormal expressions of specific miRNAs have been found to be associated with metastasis and invasion of NPC cells [14]. Moreover, EMT plays key roles in the early stages of metastatic progression, and is characterized by the loss of epithelial markers (such as E-cadherin and α-catenin) and gain of mesenchymal markers (such as Snail-1, N-cadherin, fibronectin and Vimentin) [36, 37]. Previous studies suggested that numerous miRNAs function in EMT of cancer cells, such as miR-9 and miR-23a [38, 39]. EBV-miR-BART7-3p promotes EMT and metastasis of NPC cells by repressing the tumor suppressor PTEN, as reported by Cai et al. [40]. Yue et al. have reported that EMT plays an important role in cervical LNM in nasopharyngeal carcinoma [41]. In the current study, both over-expression of miR-506 and silencing of LHX2 were detected to elevate the level of E-cadherin, while inhibiting the levels of Wnt1, β-catenin, Vimentin, and Twist. Collectively, the current study demonstrated that EMT and LNM were remarkably suppressed as a result of up-regulation of miR-506 or silencing of LHX2 in contributing to the treatment of NPC.

RETRACTED

One of the most central findings of the current study was that miR-506 was poorly expressed while LHX2 was expressed at high levels in NPC. Moreover, our results demonstrated that either up-regulation of miR-506 or silencing of LHX2 contributed to suppression of NPC cell proliferation, migration and invasion, and induction of apoptosis, as evidenced by increased percentage of cells in the G1 phase and enhanced protein levels of cleaved caspase-3. Similarly, in line with the current findings, a previous study reported that miR-506 is down-regulated in NPC cell lines and tissues, and functions as a tumor suppressor miRNA in NPC, suppressing cell proliferation, colony formation and invasion [16]. In addition, some miRNAs have been demonstrated to exert their effects on tumor progression by regulating the cell cycle [42, 43]. Ectopic over-expression of miR-506 resulted in declining rates of esophageal cancer cell proliferation as well as an induction of arrested cells at the G1 phase, which demonstrates the role of miR-506 as a proliferation suppressor in esophageal cancer through targeting cAMP responsive element binding protein 1 [44]. In pancreatic tumor cells transfected with miR-506 mimic, an increased activating cleavage of poly (ADP-ribose) polymerase and Caspase-3 induced by gemcitabine was previously revealed, confirming the elevating effect of miR-506 on cell apoptosis [45]. In line with the bioinformatics analyses, LHX2–3’-UTR was found in this study to be a specific binding site of miR-506 which could down-regulate LHX2 gene expression after transcription. LHX2, a member of the LIM homeobox family of proteins, is implicated in the regulation of cell differentiation and proliferation, functioning in embryogenesis, and is implicated in the pathogenesis of various human cancers including gastrointestinal cancer, pancreatic cancer, breast cancer and kidney cancer [46]. Moreover, the promoted cell proliferation in vitro/vivo as well as elevated β-catenin levels was demonstrated to be resulting from or be associated with up-regulated LHX2 in pancreatic ductal adenocarcinoma [47]. Furthermore, LHX2 was observed to be capable of disrupting the activation of the Wnt/β-catenin signaling pathway and additionally, the signaling pathway can bind with TCF4 to regulate the growth and apoptosis of tumor cells [31, 32]. Previous evidence also revealed that TCF4 was a direct target of LHX2 in keratinocytes, and LHX2 positively regulated TCF4 [22]. Inhibition of the Wnt/β-catenin signaling pathway was demonstrated to be responsible for the suppression of EMT as well as the proliferation, migration and metastasis of NPC cells [48]. Our findings revealed that LHX2 is involved in NPC cell proliferation, apoptosis, invasion and migration, thereby allowing us to contemplate the possibility that miR-506 may affect NPC carcinogenesis and progression by targeting LHX2, further improving our understanding of the tumor-promoting mechanism of LHX2.

RETRACTED

In the current study, miR-506 was suggested to be involved in inhibiting the activation of the Wnt/β-catenin signaling pathway by down-regulating LHX4, by means of which the EMT-related signals were inhibited. It has been suggested that LHX2 plays a pivotal role in various epithelial-mesenchymal interactions [49]. Multiple signaling pathways, including the nuclear factor kappa B, EGFR, Wnt and transforming growth factor-β (TGF-β) signaling pathways, are involved in the regulation of EMT and LNM [50–53]. Recently, Wnt/β-catenin, widely regarded as the key pathway for carcinogenesis, was reported to play a critical role in the induction and maintenance of EMT and LNM [54]. Interestingly, dysregulated signaling of the Wnt/β-catenin signaling pathway enhances the malignancy of many human cancers, including NPC [55]. In the current study, we observed that miR-506 mimic and siRNA-LHX2 decreased the protein and mRNA expressions of Wnt1 and β-catenin. LHX2 simulated β-catenin activation is suggested to be demanded for oncogenic effects of LIM domain only 1 in pancreatic ductal adenocarcinoma [47]. YPEL3, an important tumor suppressor in NPC, reduces the expression level of Wnt mediators, causing decreased Wnt activity and β-catenin destruction [48]. Similarly, Hu et al. have reported that up-regulated LHX6 expression decreases the expression level of β-catenin in breast cancer cells, and LHX6 inhibits growth and invasion of breast cancer cells via suppression of the Wnt/β-catenin signaling [31]. Likewise, LHX8_enh1 (one of the enhancers located upstream of LHX8) is also proved to be a direct target of the Wnt/β-catenin signaling [56].

## Conclusions

Altogether, the current study demonstrates that miR-506 functions as a tumor suppressor and represses EMT and LNM in NPC by inhibiting the expression of LHX2, accompanied by declining TCF4 (Fig. 13). The mechanism of miR-506 targeting LHX2 in the carcinogenesis and progression of NPC involves the Wnt/β-catenin signaling, but the underlying correlations need further intensive studies due to the limited simple size and experimental conditions. Although miRNA-based therapeutic methods are still in their infancy, our findings on miR-506 are encouraging, and indicate towards a potential treatment target for NPC in the future.

RETRACTED

**Fig. 13:** miR-506 inhibited the expression of LHX2, which hampered TCF4 expression and inactivated the Wnt/β-catenin signaling pathway, consequently inhibiting tumor growth and metastasis in NPC

## Additional file

Additional file 1: **Table S1.** The STR profiling of CNE1 cell line and CNE2, 5-8F, HONE-1 and 6-10B cell lines. (DOCX 16 kb)

## Abbreviations

ANOVA: One-way analysis of variance
DMEM: Dulbecco’s modified Eagle’s medium
ECL: Enhanced chemiluminescence
EDTA: Ethylenediaminetetraacetic acid
EMT: Epithelial-mesenchymal transition
FBS: Fetal bovine serum
GAPDH: Glyceraldehyde-3-phosphate dehydrogenase
GEO: Gene expression omnibus
GFP: Green fluorescent protein
HE: Hematoxylin-eosin
HEPES: Hydroxyethyl piperazine ethanesulfonic acid
HRP: Horse radish peroxidase
IgG: Immunoglobulin G
LHX2: LIM Homeobox 2
LNM: Lymph node metastasis
miRNAs: MircoRNAs
MTT: 3-(4,5-dimethyl-2-thiazolyl)-2,5-diphenyl-2-H-tetrazolium Bromide
MUT: Mutant-type
NPC: Nasopharyngeal carcinoma
OD: Optical density
RIPA: Radio-immunoprecipitation assay
RLU: Relative luciferase activity
RT-qPCR: Reverse transcription-quantitative polymerase chain reaction
TGF-β: Transforming growth factor-β
TNM: Tumor node metastasis
WT: Wide-type
